The article "Transgenic Biofortification of the Starchy Staple Cassava (Manihot esculenta) Generates a Novel Sink for Protein" was retracted in 2012. Reasons: results that could not be reproduced; concerns about the data; concerns about the results or conclusions.

# Transgenic Biofortification of the Starchy Staple Cassava (*Manihot esculenta*) Generates a Novel Sink for Protein

**DOI:** 10.1371/journal.pone.0016256

**Published:** 2011-01-25

**Authors:** Mohammad Abhary, Dimuth Siritunga, Gene Stevens, Nigel J. Taylor, Claude M. Fauquet

**Affiliations:** 1 International Laboratory for Tropical Agricultural Biotechnology, Donald Danforth Plant Science Center, St. Louis, Missouri, United States of America; 2 Department of Biology, University of Puerto Rico-Mayaguez, Mayaguez, Puerto Rico; 3 University of Missouri-Delta Center, Portageville, Missouri, United States of America; University of Melbourne, Australia

## Abstract

Although calorie dense, the starchy, tuberous roots of cassava provide the lowest sources of dietary protein within the major staple food crops (*Manihot esculenta* Crantz). (Montagnac JA, Davis CR, Tanumihardjo SA. (2009) *Compr Rev Food Sci Food Saf* 8:181–194). Cassava was genetically modified to express zeolin, a nutritionally balanced storage protein under control of the patatin promoter. Transgenic plants accumulated zeolin within *de novo* protein bodies localized within the root storage tissues, resulting in total protein levels of 12.5% dry weight within this tissue, a fourfold increase compared to non-transgenic controls. No significant differences were seen for morphological or agronomic characteristics of transgenic and wild type plants in the greenhouse and field trials, but relative to controls, levels of cyanogenic compounds were reduced by up to 55% in both leaf and root tissues of transgenic plants. Data described here represent a proof of concept towards the potential transformation of cassava from a starchy staple, devoid of storage protein, to one capable of supplying inexpensive, plant-based proteins for food, feed and industrial applications.

## Introduction

Cassava (*Manihot esculenta*) is cultivated throughout the tropics and is a major staple food crop across tropical sub-Saharan Africa [1]. In a previous study [2], we established that the starchy roots of cassava contain no storage proteins, possess levels of total protein in the range 0.7 to 2.5% dry weight (dw) (compared to 7 to 14% in cereals [3]) and are almost completely devoid of sulfur-containing amino acids [4]–[6]. Insufficient protein intake is a major causal factor of protein energy malnutrition (PEM), which is estimated to affect one in four of the world's children [7]. With the lowest protein∶energy ratio (P∶E) of any staple food, resource-poor populations that rely on cassava as their major source of calories are at high risk of PEM [8] and developing conditions such as Kwashiorkor [9] and related pathological disorders [10].

Few reports exist of successful transgenic modification of starchy storage organs to accumulate storage proteins. Chakraborty *et al.* (2000) [11] achieved a 40% increase in the protein content of potato tubers to reach 10 to 14% dw, by accumulation of the seed albumin protein from *Amaranthus*. The protein content of sweet potato tubers was enhanced two- to threefold to obtain 12% dw by expression of the artificial storage protein ASP1 [12] but this occurred in a non-specific manner, with similar levels of artificial protein also accumulated in the transgenic shoot tissues. When the same ASP1 gene was expressed in cassava under the control of the CaMV 35S promoter [13], no increase in protein content was achieved in the storage root organs.

In the present study, cassava was genetically modified using the patatin promoter [14] to direct transgenic expression of zeolin to the tuberous roots. Zeolin is a fusion product between phaseolin, the major storage protein in common beans (*Phaseolus vulgaris*), and a truncated gamma-zein protein from maize (*Zea mays*), which directs the fused polypeptide to form stable protein bodies within the ER [15]. Previous reports have shown expression of zeolin to result in significant accumulation of this storage protein in leaf tissues of tobacco and alfalfa [16]. We report here production of transgenic cassava plants expressing zeolin in which storage roots accumulated up to 12.5% dw protein, a greater than fourfold increase compared to controls with no associated accumulation of the protein product in leaf tissues. Analysis of transgenic plants grown under greenhouse and field conditions have confirmed that this trait is stable when plants are propagated vegetatively, it does not impact plant development and it was correlated with a significant reduction in the cyanogen content of both leaf and root tissues.

## Results

### Production and analysis of transgenic plants

Cassava plants were genetically transformed with pILTAB601 and pILTAB600, in which zeolin is expressed under the control of the CaMV 35S and patatin promoters respectively. A total of 210 *in vitro* regenerated plantlets were screened, from which a subset was indentified possessing one to two copies of the zeolin transgene (Figure S1). Eleven low copy transgenic lines, seven driven by the patatin promoter and four by the 35S promoter expressing zeolin at the RNA level, were transferred to soil in pots and grown in the greenhouse to produce storage roots.

Total protein was extracted from peeled storage roots at 8 weeks after planting and every 30 days thereafter, and levels determined by Bradford assay. All seven transgenic lines in which the patatin promoter drove zeolin expression, had accumulated 9.75% to 10.60% dw protein within their storage roots by six months after planting, a 3.0- to 3.5-fold increase compared to controls (Figure 1A). Total protein content accumulated at slightly different rates between the transgenic lines (Figure 1B), but was not correlated with RNA expression levels (Figure S1C). When total protein extract was loaded on an SDS gel, strong bands corresponding to the size of zeolin were found at significantly higher levels in transgenic storage root tissues than in leaves (Figure 1C). Conversely, plants in which zeolin expression was driven by the 35S promoter showed no significant increase in protein content of storage roots (Figure 1A) as determined by Bradford assay. In these plants presence of zeolin was observed in leaf extracts but barely detectable in storage root tissues (Figure 1C) when expressed under this constitutive promoter. Western blotting with antibodies specific to the phaseolin component confirmed presence of zeolin in the respective tissues (Figure 1D).

**Figure 1:** Protein accumulation in leaves and peeled storage roots of transgenic cassava expressing zeolin under control of the patatin and 35S promoters. **A**) Protein content in storage roots as quantified by Bradford assay after 7 months of growth in pots in the greenhouse. Non-transgenic cassava cv. 60444 (dark green bar) and transgenic plant line with empty gene vector only (pCambia2300) (light green bar) show total protein content of less than 3% dw, while all seven transgenic lines expressing zeolin under control of the patatin promoter (blue bars) accumulate total protein at 9.5% to 10.3% dw. Storage roots from plants expressing zeolin under control of the 35S promoter (orange bars) do not accumulate protein at levels above controls. **B**) Accumulation of total protein in peeled storage roots of pot grown transgenic plants expressing zeolin under control of the patatin promoter with time, as assessed by Bradford assay. Total protein content of non-transgenic cassava cv. 60444 (green bar) shows no increase over a 7 month cultivation period in the greenhouse, while the three transgenic events studied accumulated protein at slightly differing rates, but all reached approximately 10% dw by the end of the 7 month period. **C**) SDS-PAGE of crude protein extracted from leaves and roots of *in vitro* transgenic cassava lines expressing the zeolin transgene. Forty micrograms of protein extract were loaded as follows: lane 1: protein ladder; lanes 2 and 3: non-transgenic cassava cv. 60444 leaves and roots respectively; lanes 4 and 5: leaves and roots of transgenic cassava line transformed with pILTAB601 in which 35S drives expression of zeolin; and lanes 6 and 7: leaves and roots transgenic cassava line transformed with pILTAB600 in which the patatin promoter drives expression of zeolin. Presence of distinct band at 65 kDa in transgenic plants, but not in the control, indicates accumulation of zeolin in leaves of plants transgenic for 35S-zeolin and roots of plants transgenic for patatin-zeolin, but not *vice versa*. **D**) Western blot analysis of leaves (L) and peeled storage roots (R) harvested from greenhouse soil beds at 7 months of age. Total protein was isolated, 100 µg loaded in each lane and detected with specific anti-zein antibodies. Presence of zeolin protein was detected in all tissues, but accumulated at 3.5 times greater amounts in roots when expressed under the control of patatin versus the 35S promoter with the reverse pattern seen in leaves. **E**) Immuno-printing of 50–100 µm thick sections of cassava storage roots from transgenic line pILTAB600-25 in which the patatin promoter drives zeolin. Plants were grown in pots in the greenhouse and harvested from one to sevens months of age with non-transgenic cv. 60444 used as a control (top right panel). Presence of zeolin is clearly seen in roots of all ages in the transgenic, but not the control root sections, with significant accumulation in the core (xylem parenchyma) as well as the outer peel layer. Bars = 1 cm.

Immunoprinting of cassava storage roots further indicated that the transgenically expressed zeolin accumulated within both peel and xylem parenchyma storage tissues of tuberous roots (Figure 1E), while immunofluorescence studies revealed sub-cellular localization of zeolin within novel, globular protein bodies distributed within xylem parenchyma cells of 10-week-old storage roots (Figure S2). These structures were isolated by Ficoll gradient allowing identification of spherical bodies, 5 to 7 µm in diameter under the scanning electron microscope (Figure S2). No such structures were observed in non-transgenic controls and have never previously been reported within tissues of this species.

### Accumulation of storage protein and performance of fully-grown cassava plants

Three transgenic lines in which zeolin was driven by the patatin promoter were planted in soil beds in a greenhouse to facilitate production of mature plants. Total protein content within peeled storage roots harvested from these plants at 7 months of age reached 10 to 11% dw in all three transgenic lines tested (Figure 2A). Plants of the same lines, plus one in which zeolin was under control of the 35S promoter, were also established in the field at the University of Puerto Rico (Mayaguez) and assessed for agronomic characteristics and protein content of the storage roots at 11 months of age. No morphological differences were observed between transgenic and non-transgenic plants and no significant differences were apparent for average shoot or root yields, harvest index or dry matter and starch content of tuberous roots harvested from transgenic and control plants (Figure 2C) (Figure S3). Total protein content of field grown, peeled storage roots in which zeolin was driven by the patatin promoter reached 11.9 to 12.5% dw, a 4.1- to 4.3-fold increase compared to non-transgenic controls. As observed in greenhouse grown plants (Figure 1A), no increase in total protein content was detected in roots in which zeolin was under control of the 35S promoter (Figure 2A).

**Figure 2:** Characterization of fully-grown zeolin expressing plants. **A**) Total protein content of peeled storage roots harvested from transgenic cassava plants expressing zeolin grown in greenhouse soil beds and in the field. Non-transgenic plant 60444 (green bar); plant line transgenic for empty gene vector control (pCambia2300) (light green bar); plants transgenic for patatin promoter-zeolin (pILTAB600; blue bars); plants transgenic for 35S promoter-zeolin (pILTAB601; orange bar) n = 7. Assessment of total protein content by Bradford assay of storage roots shows similar results from both locations with non-transgenic, empty vector control and 35S driven zeolin varying from 2.9 to 3.1% dw, and all three events transgenic for patatin driven zeolin accumulating 3 to 4 times this amount of total protein. Total protein content from roots of field-grown plants was higher in all three lines compared to greenhouse-grown, with maximum levels of total protein reaching 12.3% dw in line pILTAB600-25. **B**) Evaluation of important agronomic traits of zeolin expressing cassava plants grown for 11 months in the field in Puerto Rico. Non-transgenic cv. 60444 plant line (green bar), plant line transgenic for empty gene vector control (pCambia2300) (light green bar), plants transgenic for patatin promoter driven zeolin transgenic lines (pILTAB600) (blue bars); plants transgenic for 35S promoter driven zeolin (orange bar) n = 12. Transgenic events showed no significant differences compared to controls across traits studied.

Western blot analysis was performed on flour extracted from 7-month-old field grown, peeled storage roots and leaf tissues. As observed from greenhouse grown plants, zeolin was found to be present in both organ types but in significantly higher amounts in transgenic storage roots compared to leaves of the same plant when patatin was the promoter employed to drive transgene expression. Use of the 35S promoter produced the opposite effect, with little accumulation in the roots but significant presence of transgenically derived protein in the leaves (Figure 1C).

### Amino acid profile and forms of accumulated zeolin

Peeled storage roots were collected from 7-month-old plants of the patatin driven zeolin-expressing line pILTAB600-25 grown in greenhouse soil beds and analyzed to determine amino acid composition. Levels of total (free+bound) amino acids increased in transgenic roots (from 3.67% to 11.87% dw) to reach 3.5 to 4.0 times that of non-transgenic controls (Figure 3A), amounts closely corresponding to the total increase in protein content. Conversely, levels of free amino acids were found to be reduced approximately threefold (from 0.62% to 0.22% dw) in these tissues compared to wild type controls. Unlike non-transgenic plants, the most abundant free amino acids detected in transgenic cassava were Aspartate and Glutamate (Figure 3A), both of which are known to be forms of nitrogen transport in cassava [17].

**Figure 3:** Analysis of amino acid and cyanogenic content in cassava tissues transgenic for zeolin. **A**) Total amino acid profile of storage roots of non-transgenic cassava cv. 60444 (green bars) and transgenic line pILTAB600-25 (blue bars) in which zeolin is driven by the patatin promoter. Increase in amounts of individual amino acids in transgenic root tissue varied from a four- to ninefold increase compared to the non-transgenic control in a manner that reflects the expect amino acid profile for zeolin. **B**, **C**) Levels of cyanogens present in cassava leaf and root tissues of seven-month-old, pot grown plants. All transgenic lines showed a reduction in cyanogen content within leaves and storage roots compared to the non-transgenic control and was apparent in transgenic events in which zeolin was under control of either the patatin (pILTAB600, blue bars) or 35S (pILTAB601, orange bars) promoters. A maximum reduction of 55% was observed in roots of pILTAB600-25, the transgenic event that accumulated the highest levels of total protein within its storage roots.

Compositional analysis of total amino acids revealed levels of individual amino acids reflecting that of zeolin, such that all essential amino acids (except tryptophan, which is absent in zeolin) were enhanced 4- to 9-fold in transgenic cassava roots (Figure 3A). Importantly, the sulfur-containing amino acids cysteine and methionine, known to be very low in cassava [4], were elevated 9- and 4.5-fold respectively in zeolin-expressing roots as compared to non-transgenic control tissues (Figure 3A). Considering that total protein content increased from ∼3% to 11% dw in this transgenic line (Figure 2A), six amino acids (Asp, Glu, Val, Met, Leu and Phe) showed a 100% match with the calculation for this level of zeolin, while Thr, Ala, Cys and Lys increased by more than 120% (Figure 3A). This data indicates that the modified total amino acid profile can be largely accounted for by accumulation of zeolin, but also in a minor way by the presence of other cassava proteins. While micro-Kjeldahl nitrogen results showed that total nitrogen content increased from 4.3% to 12.1% (2.8×) in the roots of transgenic plants grown in soil beds, Bradford assay measurements showed that the protein content was elevated from 3.0% to 11.3% (3.8×) in the roots of the same transgenic plants.

Further studies were carried out on the nature of the accumulated zeolin and associated proteins. Western blot analysis was performed on crude protein extracted from peeled storage roots of greenhouse grown, transgenic cassava. Four distinct forms of zeolin were observed (Figure S2), and respective levels of abundance determined by band intensity. Approximately 6% of the total zeolin was found present as a monomer, 76% as a trimer, 14% as a trimer bound to BiP chaperone, and 4% in a higher molecular weight, glycosylated form [16], [18]. When protein bodies were isolated without a reducing agent and loaded onto a native polyacrylamide gel, band patterning showed a higher molecular weight than expected for zeolin (Figure S2), once more suggesting that other proteins were associated with the transgenically expressed product. This high molecular weight band was eluted, sonicated and loaded onto a SDS-PAGE denaturing gel, allowing detection of proteins at different sizes, ranging from 15–90 kDa (Figure S2). The 90 kDa band was digested and confirmed by MS-ID to consist of zeolin protein, BiP chaperone and ER resident ATPases, while smaller bands contained precursor proteins, including rubisco precursors, ATPases precursors and ER membrane proteins (Table SI). To determine whether zeolin was associated with folding chaperones, an ATP-affinity assay was performed on crude proteins extracted from transgenic storage roots. Results showed that zeolin was present tightly linked to BiP chaperone in the transgenic cassava root tissues (Figure S2).

### Impact of transgenically accumulated protein on cyanogenic glycoside content

Cassava is well known as a crop species that generates and stores cyanogenic glycosides within its tissues [17], [19], [20]. Greenhouse grown plants were analyzed to determine if accumulating transgenically derived storage protein would impact the cyanogenic glycoside content of such plants. Analysis of zeolin expressing plants using an Orion CN-sensitive electrode, revealed a reduction in cyanogenic content in both leaves and storage root tissues of up to 55% compared to non-transgenic control plants (Figure 3B). Cyanogen reduction was observed in all transgenic lines and occurred when both patatin and 35S promoters were used to drive zeolin expression.

## Discussion

Although an excellent source of carbohydrate, storage roots of cultivated cassava contain only 2–3% dw protein [21]. Modifying this large storage organ to become a sink for protein through conventional methods is significantly constrained by lack of naturally occurring germplasm with high protein content and the complexity of cassava breeding programs [22]. Transgenic approaches are therefore an attractive method for directing accumulation of nutritionally balanced, or industrially valuable protein to these large storage organs. The present study was initiated to demonstrate capacity to transgenically modify cassava to accumulate storage protein of known amino acid profile within the tuberous roots. While the zeolin product described here is not intended for release to African farmers, the results described represent a proof of concept towards the potential transformation of cassava from a starchy staple, devoid of storage protein [2], to one capable of supplying both calories and nutritionally balanced proteins at dietary significant quantities to those dependent on the crop.

Zeolin expression in cassava under control of the patatin promoter caused *de novo* formation of protein bodies in storage root cells in a manner never previously reported within tissues of this species (Figure S2B), and resulted in an increase in total protein content of approximately fourfold to reach 12.5% dw (Figure 2A). Detailed analysis of these protein bodies confirmed that they consisted of different forms of zeolin and carried the nutritionally valuable, amino acid profile of the predicted storage protein, in this case phaseolin (Figure S2C, D, E).

When commencing this work there was concern that modification of cassava to accumulate significant levels of storage protein in the starch-rich storage roots would not be stable and/or would lead to disrupted physiology and altered phenotype of the transgenic plants. Greenhouse and field studies revealed this not to be the case, with similar levels of protein accumulation recorded across more than three years of testing in three different locations (Figure S3A, C, E). In addition, agronomic characteristics of the transgenic plants determined during confined field trials, showed no significant changes compared to control plants (Figure 2B). A significant pleiotropic effect of zeolin expression was seen, however, as a correlated reduction in free amino acid levels and cyanogen content in transgenic plants (Figure 2B, C). Cyanogenic levels, considered by some to be a food safety concern in this crop [10], were reduced by up to 55% in both leaf and storage root tissues and occurred when both the 35S and patatin promoters were used to drive zeolin expression.

Earlier work to enhance the nutritional quality of cassava storage roots [13], expressed the storage protein ASP1 [23] under control of the 35S constitutive promoter, but the resulting plants did not accumulate protein within their tuberous roots [24]. Likewise, in the present study, when the constitutive 35S promoter was used to drive expression of the transgene (Figure 2C, D), total protein content of root storage organs was never significantly elevated above that of the non-transgenic controls (Figures 1A & 2A). This finding indicates that the use of a suitable promoter is required to achieve accumulation of protein products in cassava storage roots. Cassava storage roots are not tubers but modified roots, which have evolved to store starch within proliferated xylem parenchyma. Considered sink specific with high activity in root tissues [14], the Class II patatin promoter used in this study was found to drive expression of zeolin RNA in leaves at levels approximately 50% of that detected in cassava storage root tissues (Figure S1C). Accumulation of the zeolin protein when derived under the control of the patatin promoter was, however, almost totally restricted to the storage roots, and remained at very low levels in leaf tissues (Figure 1C & 1D). We hypothesize, therefore, that the observed promoter-dependent, organ specific accumulation of zeolin may result, at least in part, from source/sink partitioning of nitrogen resources between the leaves and storage roots. For example, reduced levels of cyanogen of up to 55% within leaf tissues, when zeolin was expressed by either the 35S or patatin promoter, supports previous evidence that a flow of cyanogens exists between leaves and storage roots in cassava [17], [19], [20]. Furthermore, micro-Kjeldahl results showed that the total nitrogen increased by three folds in the roots of the transgenic plants and the total amino acid analysis showed that glutamate and aspartate were abundant in the storage roots of zeolin expressing plants. The difference between micro-Kjeldahl (3×) and Bradford assay measurements of the total protein content (4×) is due to the non-proteinaceous nitrogen content in cassava. Studies are ongoing to determine if this non-proteinaceous nitrogen pool, which is unique among the major crop species, is being utilized to support synthesis of storage protein in the tuberous roots of transgenic cassava plants, and if growth under conditions of differing soil nitrogen availability can affect levels of storage protein accumulation.

Cassava has the lowest protein∶energy ratio (P∶E) of any staple food, with protein content ranging from 1 to 3% dw. Thus, a two-year-old child consuming 50% of his/her dietary energy as wild type cassava will receive about 5 g dietary protein, equivalent to 35% of their daily protein requirement. The same child consuming the same amount of modified cassava accumulating storage protein at levels achieved in the present study would obtain approximately 18 g of dietary protein, or more than 100% of their daily requirement. This illustrates that genetic modification of cassava could be a potentially important component of delivering enhanced nutrition to at-risk populations in the tropics.

Accumulation of storage protein in transgenic cassava to the levels achieved in this study was not limited by a capacity to synthesize particular amino acids, which were elevated between 4.5 and 11 times compared to that of wild type, and in a manner that reflected the amino acid profile of zeolin (Figure 3B). Cassava storage roots provide a large harvest index with reported yields of up to 70 tons/ha [4], translating to a potential of 2.9 tons/ha protein product at the 12.5% dw levels achieved here. Demonstrated capacity to modify this large organ into a novel sink for nitrogen indicates that cassava likely possesses significant potential to produce and accumulate a range of proteins with nutritional, industrial or pharmaceutical value in a manner that deserves further investigation.

## Materials and Methods

### Plasmid construction

The chimeric zeolin gene was amplified from its original vector, using primers ZaF:5′AGATCTATGATGGAGCAAGGGTTCC3′ and ZeR:5′AGGTACCCTGTTTGTTGATCAGCTTC3′, with *BglII* and *KpnI* restriction sites designed within the primer sequence. The PCR product was cloned into pGEM-T vector (Promega), sequenced, the inserted fragment digested with *Bg*lII and *Kpn*I and cloned downstream of the CaMV 35S or the Class II patatin promoter. Cassettes comprising promoter-zeolin-tNOS were cloned into the pCambia2300 binary vector (http://www.cambia.org/daisy/bioforge_legacy/3724.html), to generate pILTAB600 for patatin promoter and pILTAB601 for 35S promoter versions respectively.

### Plant transformation and selection of transgenic lines

*Agrobacterium tumefaciens* strain LBA4404 harboring pILTAB600 and pILTAB601, and pCambia2300 as a control were used to genetically transform cassava friable embryogenic callus of the West African cultivar 60444 [25]. Transformed cells were recovered, and plants regenerated on selection media, propagated and sampled for DNA, RNA and protein analysis. DNA was extracted from leaves of *in vitro* plants according to the Dellaporta method [26] and used for PCR and Southern blot analysis. In the latter, 10 µg of DNA were digested with *Bg*lII or *Bg*lII+*Kpn*I, loaded on a 0.8% w/v agarose gel, transferred onto N+ Hybond membrane (GE Healthcare) and hybridized with a non-radioactive probe for the zeolin gene, prepared using the AlkPhos kit (GE Healthcare). Extraction of RNA from transgenic events was performed from *in vitro* plants and from 7-month-old plants grown in the greenhouse at DDPSC using Trizol reagent according to the manufacturer's instructions. First strand cDNA was generated using the Superscript II system (Invitrogen) from 1 µg of RNA template and subsequent PCR performed using 1 µg of cDNA and zeolin primers ZeF and ZeR. Northern blots were performed by loading 10 µg of total RNA onto 1% w/v formaldehyde agarose gel, transfered to N+ Hybond membrane and hybridized using a AlkPhos non-radioactive DNA probe generated from the zeolin sequence. RNA levels were determined using ImagQuant software to measure band intensity.

### Greenhouse growth conditions

Transgenic cassava events with low (1 to 2) copy number, high RNA expression and high protein content were propagated and transferred to soil in 7 cm pots grown in the greenhouse, and evaluated for protein accumulation. Supplemental lighting was provided for 14 hours daily with 1000 W metal halide fixtures. Artificial lights provided an average photosynthetically active radiation (PAR) of 250 µmol m^−2^ s^1^. Air temperature was maintained at 28°C during the day and 25°C at night. Fertilizer was applied at 200 ppm N three times per week using Jack's 15-16-17 Peat Lite and once a week with Jack's 15-5-15 Cal-Mag.

Vegetative clones of transgenic cassava were also evaluated by planting directly into soil beds in a greenhouse. Plants were established at DDPSC in 7 cm pots and transferred when 25 cm tall to the University of Missouri Delta Research Station, Portageville, MO. The soil consisted of Tiptonville sandy loam soil (fine-loamy, mixed, thermic Typic Argiudolls), determined to contain 60 kg NO_3_-N ha^−1^, 184 kg Bray-1 P ha^−1^, and 351 kg ammonium acetate extractable K ha^−1^. Soil was mechanically tilled and cassava plants transplanted into the earth floor at 1 m spacing. Supplemental lighting was provided for 16 hours with Sun System III 1000 W metal halide lights, providing an average PAR of 1175 µmol m^−2^ s^−1^. Air temperature was thermostatically maintained at 25 to 30°C. No fertilizer was applied during this experiment.

### Confined field trials

Transgenic cassava was grown for 11 months at the Isabella Agriculture Research Station of the University of Puerto Rico, Mayaguez in Northeast Puerto Rico, in a randomized block design with 3 reps and 8 plants/line/rep. A uniform distance of 1.5 m spacing was maintained between each plant and the entire plot surrounded by a row of wildtype 60444 plants. All steps to confine and contain the transgenic material were observed as regulated by USDA APHIS. Yield data comprising the number of roots above and below ground mass were measured per plant at harvest, 11 months after planting. Dry matter content and starch content were calculated by computing specific gravity *X* per plant root, where *X* = W_water_/(W_air_−W_water_). W_air_ is normal weight of 3 to 5 kg of roots while W_water_ is the weight in water of those same roots. Dry matter percentage and starch percentage is then equal to 158.3*x*−142 and 112.1*x*−106.4, respectively [27]. Harvest index was calculated by assessing the proportion of root fresh weight as a ratio of the total fresh weight of the plant [28].

### Immuno-fluorescence and immuno-printing

Sections of peeled cassava storage roots 50 to 100 µm thick were obtained from 10-week-old plants grown in DDPSC greenhouses in 7 cm pots. Sections were fixed in 4% para-formaldehyde and washed with TBST buffer (10 mM Tris-HCl, pH 7.5, 150 mM NaCl, 0.05% Tween 20). Fixed cells were treated with cell wall lysing enzyme Drisalase (Sigma) for 15 min, washed five times with TBST, incubated with anti-phaseolin antibodies for one hour, washed five times with TBST and incubated again with Alexa-Fluor 488 fluorescent secondary antibodies (Invitrogen) for another hour. Cells were washed five times with TBST buffer and spread on glass slides for visualization under the confocal microscope (Nikon Eclipse E-800 C1) with 100 ms exposure.

For immunoprinting, the same storage roots were washed with sterile water, cut into 1 to 3 mm thick sections, squashed onto nitrocellulose membrane and allowed to dry at room temperature. The membrane was blocked with 5% v/v skimmed milk and hybridized with anti-phaseolin antibodies, washed five times with TBST buffer and incubated with HRP secondary antibodies for an hour at room temperature. The signal was developed after washing with TBST buffer and exposing the membrane to X-ray film.

### Micro-Kjeldahl and amino acid analysis

The nitrogen content and amino acid composition of transgenic line pILTAB600-25 was compared with non-transgenic roots collected from 7-month-old soil bed grown plants. Harvested cassava storage roots were peeled, sliced into pieces 1 cm thick, lyophilized and ground into fine powder using a coffee grinder. The amino acid composition of flour produced from transgenic and non-transgenic cassava was analyzed by the Dept. of Chemistry, University of Missouri, Columbia, MO by Chemical analysis, AOAC Official Method 982.30 E (a,b,c), chp. 45.3.05, 2006.

### Protein extractions and Western blot analysis

Storage root samples were cut into 1 cm cubes, dried using a freeze-dryer and crushed into powder with a pestle and mortar. Total protein was extracted from dry samples collected at different growth stages according to Mainieri *et al* [15], and quantified by Bradford assay. A 100 mg tissue sample was placed in a 2 ml tube with a ceramic bead, 1 ml of protein extraction buffer and homogenized using FastPrep machine (MP Biomedicals). The homogenate was filtered through layers of cheesecloth, protein precipitated with TCA and quantified. Equal protein concentration were loaded on a 12% w/v polyacrylamide gel and blotted onto a nitrocellulose membrane for Western blot analysis. Anti-phaseolin primary antibodies were used after blocking the membrane with 5% skimmed milk in TTBS buffer, and HRP secondary anti-bodies used for subsequent quantification after film development using ImageQuant software (GE Healthcare).

### Mass-spectrometry identification (MS-ID)

Eluted protein bands from the native (without a reducing agent or SDS) and denaturing PAGE were digested and subjected to nano-LC-ESI-MS/MS analysis. Nano-LC was performed by LC Packings Ultimate system (San Francisco, CA) equipped with a Dionex C18 PepMap100 column (75 µm i.d.) (Sunnyvale, CA) flowing at 180 nL/min. Peptides (5 µl injections) were resolved on a gradient that started at 95% solvent A (5% acetonitrile, 0.1% formic acid) and 5% solvent B (95% acetonitrile, 0.075% formic acid in MilliQ water) for 3 min, then increasing from 5 to 25% B over 5 min, from 25 to 60% B over the next 32 min, and from 60 to 95% B over the final 5 min. Mass spectrometric analysis was performed on an ABI QSTAR XL (Applied Biosystems/MDS Sciex) hybrid QTOF MS/MS mass spectrometer equipped with a nanoelectrospray source (Protana XYZ manipulator). Positive mode nanoelectrospray was generated from fused-silica PicoTip emitters with a 10 µm aperture (New Objective) at 2.5 kV. TOF mass and product ion spectra were acquired using information dependent data acquisition (IDA) in Analyst QS v1.1 with mass ranges for TOF MS and MS/MS at m/z 300–2000 and 70–2000, respectively. Every second, a TOF MS precursor ion spectrum was accumulated, followed by three product ion spectra, each for 3 s. Switching from TOF MS to MS/MS was triggered by the mass range of peptides (m/z 300–2000), precursor charge state [2]–[4] and ion intensity (>50 counts). The DP, DP2, and FP settings were 60, 10, and 230, respectively, and rolling collision energy was used.

### Determination of ATP-affinity bound proteins

Five grams of three-month-old transgenic, peeled cassava storage roots harvested from transgenic line pILTAB600-25, grown in 7 cm pots in DDPSC greenhouses, were gently homogenized in TBS buffer containing proteinase inhibitor cocktail (Sigma) and filtered using four layers of cheesecloth. Cell lysate was passed through a 22 µm filter, loaded on 5, 10, 15, and 20% Ficoll gradient and centrifuged for 3 hr at 15 000 rpm in 4°C. Precipitated proteins were collected and incubated with ATP-Sephasrose (Jena-Bioscience) to capture ATP bound proteins following manufacturer instructions. ATP bound proteins were loaded on native and denaturing acrylamide gels and protein bands eluted and identified using MS-ID. The same precipitate recovered from Ficoll was washed with TBS buffer, blotted on nitrocellulose membrane and hybridized with anti-phaseolin and secondary Alexa-fluor 488 antibodies for evaluation under the fluorescent and scanning electron microscope (Hitachi TM-1000 tabletop).

### Determination of cyanogenic content

Cassava leaf and root samples were collected from plants at six months of age growing in 7 cm pots in the greenhouse and 100 mg fresh tissue ground in a closed tube containing 1 ml TBS buffer using a FastPrep machine (MP Biomedicals). Tubes were incubated for 10 min at room temperature then placed in 50 ml closed tubes containing 9 ml of 5M NaOH. Content of cyanogenic compounds was measured using an Orion CN-sensitive electrode (Thermo-Scientific) after preparing a standard curve of KCN. The electrode sensitivity was evaluated by measuring the HCN captured in 5M NaOH from *β*-glucosidase activity on known concentrations of pure linamarin purchased from (Sigma) and processed in the same way.

## Supporting Information

Figure S1 **Transgenic nature and expression of zeolin in cassava.** **a**) PCR amplification of DNA from a subset of the 210 *in vitro* transgenic plants produced, using primer set ZeF and ZeR specific for zeolin. Non-transgenic cv. 60444 was used as a negative control and pILTAB600 plasmid as a positive control, followed by transgenic cassava transformed with genetic constructs pILTAB601 and pILTAB600. **b**) Southern blot of DNA extracted from *in vitro* leaf tissue of transgenic cassava plants. Lanes 3–11: plants transformed with pILTAB600 and lanes 12–19 plants transformed with pILTAB600. Non-transgenic cassava cv.60444 was used as a negative control and plasmid pILTAB600 as positive control. Upper panel shows DNA digested with *Bgl*II to confirm integration and copy number of the zeolin transgene, lower panel shows DNA digested with *Bgl*II and *Kpn*I to confirm intact nature of integrated sequence. **c**) Determination of zeolin RNA expression in transgenic tissues. Northern blotting was performed on 10 µg total RNA extracted from *in vitro* and seven month old greenhouse grown leaves and roots of plants transgenic for zeolin under control of the 35S (pITAB601) and patatin (pILTAB600) promoters. Expression levels were equivalent for both constructs in leaves and roots (L and R respectively) from *in vitro* grown plants, but significantly different in plants grown in the greenhouse. In the latter, the 35S promoter drove 3–4 times higher expression of zeolin in the leaves than in the roots, while patatin drove zeolin RNA expression at significantly higher levels in the roots than in leaf tissue. Transgenic tobacco leaff and root tissues were used as a positive control.
(TIF)

Figure S2 **Characterization of zeolin accumulation in roots of transgenic cassava.** a) left panel; Western blot analysis of 50 µg protein extracted without reducing agent from transgenic cassava storage roots from six different plants (clones) of transgenic line pILTAB600-25, using antibody against phaseolin. Four different forms of zeolin protein were visualized in accordance with Bellucci *et al.*, ^13^, with smallest band size representing newly synthesized zeolin polypeptide found as a monomer, zeolin trimers then zeolin trimers bound to the folding chaperone BiP. Right panel; re-probing with BiP specific antibodies confirmed binding of zeolin to BiP chaperones in cassava root tissue. **c**) Localization of zeolin accumulation as protein bodies within the xylem parenchyma of cassava storage roots. (top left panel) non-transgenic cassava storage root cells. (top right panel) cells of transgenic storage roots in which zeolin is labeled with fluorescent secondary antibody showing zeolin accumulating as discrete bodies. (lower panel) scanning electron microscopy of purified zeolin protein bodies isolated from transgenic cassava storage roots of plant line p600-25. Zeolin protein bodies range in size from 3 to 7 µm in diameter. **c**) Native PAGE of purified protein bodies isolated from storage root tissue of thee pILTAB600-25 plant lines showing signal at higher MW size than expected for zeolin (65 kDa). **d**) SDS-PAGE gel of the high MW bands from **c** after elution and sonication. All bands were eluted and analyzed by MS-ID, confirming upper band as zeolin with BiP chaperone and smaller protein bands (arrowed) as rubisco precursors **e**) ATP affinity assay for total protein extracted from transgenic cassava storage roots of pILTAB600-25. Bands were eluted and analyzed by MS-ID to identify zeolin associated with ATP chaperones, ATPase precursors and ER membrane proteins.
(TIF)

Figure S3 **Transgenic cassava plants of cv. 60444 expressing the chimeric storage protein zeolin.** **a**) Transgenic plants producing storage roots (**b**) growing in pots in the greenhouse at DDPSC **c**) Transgenic plants expressing transgenic storage protein growing in a soil bed in the greenhouse. Plants reach 3.5 m in height and produce up to 10 storage roots per (**d**) plant within six months. **e**) Transgenic plants expressing zeolin growing in confined field trial at the University of Puerto Rico, Mayaguez. Plants in the field showed no significant morphological differences to the non-transgenic controls and produced mature storage roots within 10–11 months.
(TIF)

Table S1 **Protein identity of eluted and digested protein bands from the SDS-PAGE (Figure S2D and S2E).** All bands from Figure S2D and S2E were eluted, digested, and analyzed by MS-ID as detailed in Materials and Methods. The table provides: GI Accession number for the blast result, Protein Identity, Source of the Protein, Score Identity to the aligned protein from the source organism, and Peptide Coverage percentage of the sequenced amino acids in the digested proteins compared to the source organism proteins.
(DOC)
